# Hypoxia Preconditioned Mesenchymal Stem Cells Prevent Cardiac Fibroblast Activation and Collagen Production via Leptin

This article has been retracted.

**DOI:** 10.1371/journal.pone.0103587

**Published:** 2014-08-12

**Authors:** Panpan Chen, Rongrong Wu, Wei Zhu, Zhi Jiang, Yinchuan Xu, Han Chen, Zhaocai Zhang, Huiqiang Chen, Ling Zhang, Hong Yu, Jian'an Wang, Xinyang Hu

**Affiliations:** 1 Division of Cardiology, the Second Affiliated Hospital, College of Medicine, Zhejiang University, Zhejiang Province, Hangzhou, China; 2 Provincial Key Laboratory of Cardiovascular Research, Zhejiang Province, Hangzhou, China; Georgia Regents University, United States of America

## Abstract

**Aims:**

Activation of cardiac fibroblasts into myofibroblasts constitutes a key step in cardiac remodeling after myocardial infarction (MI), due to interstitial fibrosis. Mesenchymal stem cells (MSCs) have been shown to improve post-MI remodeling an effect that is enhanced by hypoxia preconditioning (HPC). Leptin has been shown to promote cardiac fibrosis. The expression of leptin is significantly increased in MSCs after HPC but it is unknown whether leptin contributes to MSC therapy or the fibrosis process. The objective of this study was to determine whether leptin secreted from MSCs modulates cardiac fibrosis.

**Methods:**

Cardiac fibroblast (CF) activation was induced by hypoxia (0.5% O_2_). The effects of MSCs on fibroblast activation were analyzed by co-culturing MSCs with CFs, and detecting the expression of α-SMA, SM22α, and collagen IαI in CFs by western blot, immunofluorescence and Sirius red staining. In vivo MSCs antifibrotic effects on left ventricular remodeling were investigated using an acute MI model involving permanent ligation of the left anterior descending coronary artery.

**Results:**

Co-cultured MSCs decreased fibroblast activation and HPC enhanced the effects. Leptin deficit MSCs from Ob/Ob mice did not decrease fibroblast activation. Consistent with this, H-MSCs significantly inhibited cardiac fibrosis after MI and mediated decreased expression of TGF-β/Smad2 and MRTF-A in CFs. These effects were again absent in leptin-deficient MSCs.

**Conclusion:**

Our data demonstrate that activation of cardiac fibroblast was inhibited by MSCs in a manner that was leptin-dependent. The mechanism may involve blocking TGF-β/Smad2 and MRTF-A signal pathways.

## Introduction

Transplantation of bone marrow-derived mesenchymal stem cells (BM-MSCs) improves cardiac function after myocardial infarction (MI), an effect that has been attributed to a reduction in infarct size and suppression in left ventricular fibrosis [1], [2]. It has been shown that the neovascularization and anti-apoptotic effects of MSCs contribute to the improved cardiac function [3]–[5]. Anti-fibrotic effects are also implicated in the therapeutic effect of MSCs [6], [7]. However, the underlying mechanisms are incompletely understood.

Post-MI myocardial remodeling is associated with increased expression of profibrotic growth factors and activation of cardiac fibroblasts, which constitutes an important step during the post-MI remodeling process [8]. Activated cardiac fibroblasts change their phenotype and are trans-differentiated into myofibroblasts, a process that is characterized by increased expression of α-smooth muscle actin (α-SMA) and production of extracellular matrix (ECM) proteins [9]. Cardiac myofibroblasts contribute to the structural and functional changes in the heart by increasing collagen deposition, regulating autocrine/paracrine factors, and replacing of myocytes with fibrotic scar tissue [9].

The transition of cardiac fibroblasts to myofibroblasts is controlled by a variety of growth factors, cytokines, and mechanical stimuli. Transforming growth factor-β (TGF-β) is a key factor that mediates cardiac fibroblast activation and differentiation into hyper-secretory myofibroblasts. The TGF-β/Smad2 pathway is recognized as a traditional signal pathway that initiates activation of cardiac fibroblasts [10]. Recently, MRTF-A signaling was also reported to be involved in the activation of cardiac fibroblasts during post-MI remodeling [11], [12].

In our previous study, MSCs were shown to exhibit anti-fibrotic effects during post-MI remodeling process, an effect that was enhanced by HPC [1]. Other studies reported shown that exogenous leptin administration enhanced fibrosis process [13], therefore we sought to determine the precise role of leptin in the protective effects offered by MSCs. We hypothesize that leptin from MSCs is essential for inhibition of cardiac fibroblast activation; HPC of MSCs increases leptin expression, and this correlates with inhibition of cardiac fibroblast activation. Here we report that activation of cardiac fibrosis is inhibited by MSCs; the effects are enhanced by HPC and leptin plays a key role possibly by blocking both TGF-β/p-Smad2 and MRTF-A signal pathways.

## Results

### Hypoxia activates cardiac fibroblasts to myofibroblasts and increases collagen production

Transition from fibroblasts to the activated form myofibroblasts is characterized by expression of α-SMA. Fibroblasts can be activated by biochemical stimulation with TGF-β1 or Ang II [14], [15], or hypoxia treatment [16]–[19]. We confirmed that hypoxia treatment of cardiac fibroblasts increased α-SMA expression by 2.71±0.23 fold in mRNA level (H-CFs vs. N-CFs, n = 3, P<0.05) (Fig. 1 A), and 2.03±0.14-fold in protein level (H-CFs vs. N-CFs, P<0.05) (Fig. 1 B to C). A similar effect was also observed in CFs treated with TGF-β1 (Fig. 1 A to C).

**Figure 1:** Hypoxia activated cardiac fibroblasts (CFs) to myofibroblasts (MCFs) through TGF-β/Smad2 pathway and increased collagen production. Cardiac fibroblasts cultured at normoxia (N-CFs) and hypoxia condition (H-CFs), or treated with 10 ng/ml TGF-β1 at normoxia condition 24 hours (N-CFs-TGF-β1) were collected for subsequent experiments. (A) α-SMA mRNA level measured by qRT-PCR of total RNA isolated from CFs. mRNA value of H-CFs and N-CFs-TGF-β1 was normalized to N-CFs. (B) Western blots quantification of α-SMA protein expression in cell lysates from CFs after hypoxia and TGF-β1 pretreatment. The α-SMA ratios normalized to β-actin in both hypoxia and TGF-β1 treated groups were compared with the control group. (C) Representative western blot analysis of α-SMA protein expression in CFs cultured under standard condition was used as a control. Both hypoxia and TGF-β1 treatment for 24 hours increased α-SMA expression. (D) Representative western blot of collagen IαI protein expression in cell lysates from N-CFs, H-CFs and N-CFs-TGF-β1. Both hypoxia and TGF-β1 treatment for 24 hours increased collagen IαI expression. (E) Quantification of collagen IαI western blot in D. The ratios of collagen IαI normalized to β-actin in both hypoxia and TGF-β1 pretreated groups were compared with the normoxia cultured group. (F) Representative western blot of TGF-β1 and phospho-Smad2 protein expression in N-CFs and H-CFs. (G) Quantification of TGF-β1 and phospho-Smad2 western blot in F. The ratio of TGF-β1 and p-Smad2 in H-CFs were compared to normoxia cultured CFs (n = 3, *p<0.05).

Increased collagen IαI synthesis is another characteristic of fibroblast activation. Treatment of CFs with either hypoxia or TGF-β1 resulted in approximately 2.5-fold increase of collagen IαI expression (Fig. 1 D to E). It has been reported that TGF-β1/Smad2 signaling plays a crucial role during the process of cardiac fibroblast activation. Our data shows that hypoxia treatment of CFs up-regulated the expression of TGF-β1 by 4.55±0.55-fold and phosphorylated Smad by 4.02±0.54-fold in comparison with normoxia cultured CFs (P<0.05) (Fig. 1 F to G).

Taken together, these results indicate that hypoxia, like TGF-β1; can induce fibroblast transformation into myofibroblast through the TGFβ1/p-smad2 signaling pathway. Based on closely similar results of hypoxia and TGF-β1 in the activation of fibroblasts, further in vitro experiments were limited to hypoxia treatment only.

### HPC enhances suppression of Cardiac Fibroblast Activation by MSCs

Our previous study showed that hypoxia preconditioned MSCs were significantly more effective than normoxia MSCs in the reduction of infarct [1]. Because fibroblast activation and collagen synthesis are important processes in cardiac fibrosis after MI, a two-chamber co-culture system was used to determine whether HPC-MSCs convey superior inhibition of cardiac fibroblast activation.

Cardiac fibroblasts were exposed to hypoxia for 24 hours to induce activation, while MSCs were treated with either hypoxia (at 0.5% oxygen concentration 24 hours, H-MSCs) or normoxia (N-MSCs). Then CFs and MSCs were co-cultured in the two chamber assay as described in Methods, for 24 hours. Normoxia exposed CFs served as controls (N-CFs).

Compared with cardiac fibroblasts alone, co-culture with N-MSCs resulted in a significant decrease in both α-SMA (30%) and SM22α (18%) expression in the fibroblasts. An adiditional decrease in α-SMA (62%) and SM22α (35%) was observed when CFs were co-cultured with H-MSCs (N-MSCs & H-MSCs group vs. H-CFs group, P<0.05) (Fig. 2 A to B). The same pattern of changes in α-SMA was confirmed by immunofluorescence staining of CFs, showing that H-MSCs exert more inhibition of fibroblast activation in comparison with N-MSCs. (N-MSCs & H-MSCs group vs. H-CFs group, P<0.05) (Fig. 2 C to D).

**Figure 2:** H-MSCs^WT^ reverses hypoxia stimulated collagen production and cardiac fibroblast differentiation into myofibroblasts. H-MSCs^WT^ and N-MSCs^WT^ co-cultured with H-CFs at normal culture condition 24 hrs. Cardiac fibroblasts from the lower chamber which co-cultured with different preconditioned MSCs^WT^ were collected for subsequent experiments. (A) Representative western blot of α-smooth muscle actin, collagen IαI and SM22α in cellular lysates from cardiac fibroblasts co-cultured with N-MSCs^WT^ and H-MSCs^WT^. (B) Quantification analysis of western blot in A. (C) Immunofluorescence staining for α-smooth muscle actin in H-CFs co-cultured with N-MSCs^WT^ and H-MSCs^WT^. (D) Quantification analysis of images presented on (C). (E) Quantitative analysis of the effects of N-MSCs^WT^ and H-MSCs^WT^ on the collagen production induced by hypoxia in cardiac fibroblasts stained by Sirius Red, resolution in 1 mol HCl. Data are the mean ± SEM of three independent experiments. * P<0.05 versus H-CF; #P<0.05 versus H-CF-N-MSCs^WT^. Scale bars in C represent 50 µm.

In addition to suppression of α-SMA expression, N-MSCs also inhibited hypoxia-induced collagen IαI protein expression (35%) (N-MSCs group vs. H-CFs group, P<0.05) (Fig. 2 A to B) and cellular collagen accumulation (45%) detected by Sirius red staining (N-MSCs group vs. H-CFs group, P<0.05) (Fig. 2 E). As expected, a further decrease in collagen IαI protein expression (62%) and total collagen production (67%) was observed in H-CFs when co-cultured with H-MSCs compared with N-MSCs (H-MSCs group vs. N-MSCs group, P<0.05) (Fig. 2 A, B and E).

### Increased leptin expression by HPC

To identify what may be unique changes within H-MSCs, microarray assays were performed. H-MSCs exhibited a significant increase in leptin expression compared with N-MSC [20], an effect that was validated by quantitative RT-PCR assay (N-MSCs 1.00±0.17; H-MSCs: 5.49±0.20; H-MSCs vs. N-MSCs P<0.05) (Fig. 3).

**Figure 3:** Hypoxia preconditioning upregulated leptin expression of MSCs. (A) leptin mRNA level in MSCs after normoxia, hypoxia treatment were measured by qRT–PCR. Data are the mean ±SEM of three independent experiments. *P<0.05 versus N-MSC^WT^.

### Leptin-deficient H-MSCs do not prevent cardiac fibroblast activation

To test whether leptin in H-MSCs was responsible for its inhibition of cardiac fibroblast activation, MSCs from leptin deficit (ob/ob) mice (MSC^ob/ob^) were isolated and co-cultured with hypoxia-activated CFs. In contrast to the decreased expression of α-SMA and SM22α in H-CFs when they were co-cultured with H-MSCs^WT^, co-culturing with H-MSCs^ob/ob^ failed to inhibit the activation of H-CFs; SM22α 1.81±0.11 units in H-MSCs^ob/ob^ group vs. 1.11±0.07 in H-MSCs^WT^ group; α-SMA 2.50±0.10 in H-MSCs^ob/ob^ group vs. 1.67±0.15 in H-MSCs^WT^ group (P<0.05) (Fig. 4 A to B). Immunofluorescence staining of α-SMA also confirmed the lack of inhibitory effect on α-SMA expression in H-CFs by co-culturing with H-MSCs^ob/ob^ (in comparison with H-MSCs^WT^, P<0.05) (Fig. 4 C to D). A similar result was observed for collagen synthesis in H-CFs, showing lower collagen IαI mRNA expression (H-MSCs^WT^ group, 2.07±0.40 vs. H-MSCs^ob/ob^ group, 2.73±0.21, P<0.05) and less collagen protein synthesis (H-MSCs^WT^ group, 1.13±0.04 vs. H-MSCs^ob/ob^ group, 2.46±0.11, P<0.05) (Fig. 4 A, E and F). Together, these data indicate that leptin from MSCs may play a key role in regulating the activation of fibroblasts.

**Figure 4:** H-MSCs^WT^ prevent hypoxia induced cardiac fibroblast activation, but leptin deficit inhibit this effect. (A) Western blot of α-SMA, collagen IαI and SM22αin cellular lysates from hypoxia-activated cardiac fibroblasts co-cultured with H-MSCs^WT^ and H-MSCs^ob/ob^. Blots were reprobed for α-Tublin as control. (B) Quantification analysis of α-SMA and SM22α protein level expressed as % of controls (N-CFs). (C) Immunofluorescence staining of α-SMA in hypoxia-activated cardiac fibroblasts co-cultured with H-MSCs^WT^ and H-MSCs^ob/ob^. (D) Quantitative analysis of α-SMA immunofluorescence staining presented on (C). (E) Quantitative analysis of collagen protein level expressed as % of controls (N-CFs) in A. (F) Quantitative analysis of hypoxia-activated cardiac fibroblasts co-cultured with H-MSCs^WT^ and H-MSCs^ob/ob^, stained with Sirius Red. (G) Western blot of α-SMA in cellular lysates of hypoxia-activated wide type or leptin deficit db/db cardiac fibroblasts co-cultured with H-MSCs^WT^. (H) Quantification analysis of α-SMA protein level expressed as % of controls (N-CFs). * P<0.05 versus N-CF; #P<0.05 versus H-CFs-H-MSCs. Scale bars in C represent 50 µm.

To further demonstrate the key role of leptin in regulating cardiac fibroblast activation, leptin receptor deficient cardiac fibroblasts (CFs^db/db^) were isolated from db/db mice (leptin receptor deficit mice), and co-cultured with H-MSCs. As shown in Fig. 4 G and H, H-MSCs did not attenuate the activation of cardiac fibroblast from db/db mice (H-MSCs^WT^-H-CFs group, 1.75±0.31 vs. H-MSCs^WT^-H-CFs^db/db^ group, 3.01±0.07, P<0.05) (Fig. 4 G and H), indicating that effect of H-MSCs on the inhibition of CF activation is through the paracrine effect of leptin from MSCs.

### H-MSCs improved post-MI remodeling was leptin dependent

To further evaluate the role of leptin in regulating fibroblast transformation, a mouse MI model was used to compare the effects of cell therapy on the cardiac fibrosis using MSCs^WT^ vs. MSCs^ob/ob^. Infarct size at 7 days post MI was significantly decreased after transplantation of HPC MSCs^WT^ in comparison with MSCs^WT^ and PBS groups (50.05±5.35% vs. 69.08±2.82% and 77.49±0.66%, respectively; p<0.01) (Fig. 5 A and C). Such beneficial effects were absent when H-MSCs^ob/ob^ were used (72.06±3.03%, Fig. 5 A and C). Consistent with these observations, no significant difference in left ventricular collagen I expression was observed between N-MSC^WT^ therapy group and PBS group, while H-MSCs^WT^ administration resulted in a significant decrease in collagen I expression (H-MSCs^WT^ group, 5.10±0.66% vs. PBS group, 8.18±1.19%, p<0.05) (Fig. 5 B and C). Again transplantation of H-MSCs^ob/ob^ had no effect on collagen I expression (H-MSCs^ob/ob^ group, 10.78±1.92% vs. H-MSCs^WT^ & PBS group, p<0.05) (Fig. 5 B and C).

**Figure 5:** H-MSCs^WT^ reduced infarct size and collagen I expression 7 days post-MI. (A) Representative Masson's trichrome staining of heart tissue to show the infarct area (blue) 7 days after MI. (B) Representative immunofluorescence staining of collagen I (red) in LV. (C) Quantification of cardiac infarct size in A. (D) Quantification of collagen I percentage of LV in B. n = 5–6, *P<0.05 vs. others.

Myofibroblasts in the peri-infarction region were identified by FSP-1 and α-SMA positive staining. There were significantly fewer double positively stained myofibroblasts in the N-MSCs^WT^ group (38.43±2.11 unit), compared with the PBS group (58.67±3.50 unit), and the number of myofibroblasts was further reduced by transplantation of H-MSCs^WT^ (19.64±1.46 unit, p<0.05 vs. other groups) (Fig. 6 A to B). However, the beneficial effect of hypoxia preconditioning was absent when H-MSCs^ob/ob^ was used (32.00±1.82 unit).

**Figure 6:** H-MSCs^WT^ decrease myofibroblasts in peri-infarction region. (A) Immunofluorescence staining of myofibroblast (DAPI (blue), α-SMA (red) and FSP (green)) in heart frozen section. Arrows indicate double positively stained myofibroblasts. Scale bars represent 50 µm. (B) Quantification of double positive stained myofibroblasts in A, analyzed by Image Pro 6.0 software.*P<0.05 versus N-MSCs, #P<0.05 versus H-MSCs, n≥5 in each group.

### H-MSCs attenuated cardiac fibroblast activation through TGF-β1/p-Smad2 and MRTF-A pathways

To investigate the target signaling mechanisms in CFs that were affected by MSCs in the process of fibroblast activation, TGF-β1/Smad2 and MRTF-A pathways were tested. Activation of CFs by hypoxia treatment significantly increased TGF-β1, p-Smad, MRTF-A, and MRTF-B (Fig. 7 A to B). Co-culturing H-CFs with H-MSCs^WT^ abolished such up-regulation, and this was not observed by co-culturing with H-MSCs^ob/ob^ (Fig. 7 A to B). To investigate how the MRTF-A pathway in CF activation is regulated by H-MSCs^WT^, Y-27632, an inhibitor of Rho kinase, was added to co-cultures of H-CFs/H-MSCs^ob/ob^. Y-27632 inhibits the nuclear accumulation of MRTFs. We found that the nuclear accumulation of MRTF-A in CFs was induced by hypoxia, and this was inhibited by co-culturing with H-MSCs^WT^. The inhibitory effect was diminished when leptin deficient H-MSCs^ob/ob^ were used. Y-27632 inhibited the nuclear accumulation of MRTF-A (Fig. 7 C).

**Figure 7:** Leptin deficit hypoxia exposed-MSCs failed to limit cardiac fibroblast activation, through TGF-β/Smad2 and MRTF-A. (A) Western blot of TGF-β, p-Smad2, MRTF-A and MRTF-B in cellular lysates from hypoxia-activated cardiac fibroblasts co-cultured with H-MSCs^WT^ and H-MSCs^ob/ob^. Blots were reprobed for α-Tublin as a control. (B) Densitometric analysis of protein level expressed as % of controls (N-CFs). (C) Immunofluorescence staining of MRTF-A and DAPI has done in H-CFs from four groups. * P<0.05 versus N-CF; #P<0.05 versus H-CF-H-MSCs. Scale bars in E represent 50 µm.

## Discussion

Activation of cardiac fibroblasts (CFs) into myofibroblasts (MCFs) constitutes a key step during myocardial remodeling after MI, leading to heart failure. MSCs, especially hypoxia preconditioned MSCs, have been shown to attenuate left ventricular remodeling [1]. The results presented in this study confirmed that H-MSCs^WT^ exhibited significant greater effect on preventing fibroblast activation compared with N-MSCs^WT^. In addition, we showed that leptin plays a crucial role in H-MSCs-mediated inhibition of cardiac fibroblast activation, the inhibitive effects by H-MSCs were diminished when leptin was absent in H-MSCs^ob/ob^. Moreover, both TGF-β/Smad2 and MRTF-A pathways are involved in the cardiac fibroblast activation. Finally, we demonstrated that H-MSCs^WT^ improved cardiac function after MI, which was closely associated with attenuated cardiac fibrosis as evidenced by reduced fibroblast activation at the peri-infarct area, an effect that was again absent in the H-MSCs^ob/ob^ group.

The major finding of our study is that H-MSCs^WT^ inhibit hypoxia-induced cardiac fibroblast activation, while leptin deficit H-MSCs^ob/ob^ do not, indicating leptin is critically involved in the beneficial effects of H-MSCs. Previous studies have defined a dual role of fibroblasts in cardiac repair. Loss or impaired repair process by fibroblasts can lead to cardiac rupture [21] while excessive fibrosis can result in increased ventricular wall stiffness and eventually induced heart failure [21], [22]. Leptin is a 16-kDa adipokine that plays a key role in regulating energy intake and expenditure [23]. It has been shown that exogenous leptin enhances fibrosis via fibroblast activation [24], however, our present study provides novel evidence that MSCs require leptin expression to inhibit the activation of fibroblasts. Transplantation of H-MSCs^WT^ into a mouse MI model significantly reduced infarct size, alleviated collagen deposition, and thereby improved cardiac performance without showing any occurrence of cardiac rupture.

Our data indicates that endogenous leptin from MSCs functions as an antifibrotic factor. The reason behind the apparent different effects between endogenous and exogenous leptin is multi-factorial. One possible reason is that leptin may have pleitropic effects through modulating the secretion of multiple paracrine factors by MSCs, leading to a down-regulated inflammatory response, decreased infarct size and less fibroblast activation. Exogenous leptin may directly exert only its pro-fibrotic effects. We also performed microarray tests to quantify the paracrine cytokines present in the supernatant from both H-MSCs^WT^ and H-MSCs^ob/ob^. The results showed that compared to H-MSCs^ob/ob^, H-MSCs^WT^ release more anti-fibrotic proteins such as decorin, a small chondroitin–dermatan sulphate proteoglycan that exert protective effects on cardiac remodeling [25], [26]. In addition, we found that pro-inflammatory factors [27], [28], such as MIP-2, were highly secreted by H-MSCs^ob/ob^. Therefore, we suggest that the enhancement of decorin and reduction of MIP-2 secreted by H-MSCs^WT^ may be involved in inhibition of CF activation mediated by H-MSCs.

Interestingly, we also found that both TGF-β/Smad and MRTF-A signaling pathways were involved in CFs activation and were inhibited by H-MSCs^WT^. TGF-β has been identified as a primary and potent mediator of myofibroblast transformation [15], [29], and fibrotic remodeling in the heart [9]. TGF-β1 binds to its cell surface receptor and increases phosphorylation of Smad2, leading to an increased transcriptional activity, and significant upregulation of Col IαI expression [15]. Our study provides further evidence that H-MSCs inhibit CF activation partly by inhibiting TGF-β/Smad signaling. On the other hand, myocardin-related transcription factors A and B (MRTFs, MRTF-A/B) have been reported to regulate the expression of smooth muscle-specific cytoskeletal proteins, including α-SMA, in smooth muscle cells and fibroblasts [30], [31]. Our data indicates that MRTF-A/B is involved in the inhibitive effects of H-MSCs^WT^ on myofibroblast activation. Interestingly, we showed that a deficit of leptin expression of MSCs almost abolished the protective effects offered by H-MSCs, whereas the activation of MRTF-A/B was partially reversed in the leptin-deficient cells, indicating that another layer of mechanism must be involved in regulating MRTF-A signaling. This also suggests that TGF-β/Smad and MRTF-A/B signaling are the two parallel pathways that are involved in activation of CFs. Even though we showed that Y-27632, a RhoA kinase inhibitor [30], partially inhibited MRTF-A nuclear translocation, we cannot exclude the possibility that it exerts anti-inflammatory effects to down-regulate the expression of TGF-β. A further study is warranted to elucidate the relationships between these two signaling pathways.

There are some limitations that we need to address in the present study. Firstly, our data is in strikingly contrast to the published data where exogenous leptin enhanced fibrosis. Our data shows that leptin signaling is required for the protective effects especially when MSCs were hypoxia preconditioned. It warrants further investigation to determine why the differences exist between MSC-derived and exogenous leptin signaling. Secondly, even though we demonstrated that both TGF-β/Smad2 and MRTF-A play roles in activation of CFs as two parallel signaling pathways, that are attenuated by treating with MSCs, the detailed regulatory mechanisms for these two signaling were not studied. Finally, we failed to further explore whether leptin over-expression in MSCs would offer extra benefits in mediating the activation of CFs and whether there exist dose-dependent effects of leptin on TGF-β/Smad2 and MRTF-A signaling. Nevertheless, our data provide novel evidence that leptin from MSCs plays a key role in the inhibition of CF activation.

In conclusion, our data show that H-MSCs^WT^ inhibit cardiac fibroblast transformation through TGF-β/Smad2 and MRTF-A signaling and leptin signaling is mechanistically implicated (Fig. 8). Further study is needed to delineate whether a dose dependent effect of leptin exists in inhibiting fibroblast activity that might provide important evidence for its potential clinical applications.

**Figure 8:** H-MSCs^WT^ inhibited hypoxia induced cardiac fibroblast activation via leptin. Hypoxia induced secretion of TGF-β from cardiac fibroblasts, leading to Smad2 phosphorylation, meanwhile, hypoxia increased expression and nuclear translocation of MRTF-A. These two signaling pathways co-regulated the transcription of myofibroblast target gene α-SMA and collagen IαI, causing the activation of fibroblasts. Our study indicated that H-MSCs^WT^ inhibited the expression of TGF-β, phosphorylation of Smad2 and nuclear translocation of MRTF-A, leading to cardiac fibroblast inactivation, and this protective effect was leptin dependent.

## Materials and Methods

### Ethics Statement

All animal experiments were performed with approval of the Institutional Animal Care and Use Committee, Zhejiang University.

### Cardiac fibroblasts isolation and culture

Wild type C57BL/6 mice used for CFs isolation were purchased from Model Animal Research Center of Nanjing University (Nanjing, China). Mouse cardiac fibroblasts (CFs) were isolated from heart of 8–9 weeks old C57BL/6 mice. Ventricles were minced and digested in 0.05% collagenase and 0.05% pancreatin (Gibco, Invitrogen, Carlsbad, CA, USA) containing PBS solution at 37°C and waved at 220 rpm 10 min for 4–5 times. Cells were pre-plated for 1 hour on uncoated culture dishes (Corning Inc., NY, USA), during which CFs rapidly adhered to the dishes. After preplating the medium containing cardiomyocytes was removed and the attached CFs were washed and further cultured in DMEM (Gibco) containing 10% fetal calf serum (FCS, Gibco) and 10% bovine calf serum (BCS, Gibco) at 37°C and 5% CO_2_. Fresh complete medium was added and replaced every 3 days. Each primary culture was subcultured 1∶2 when CFs grew to approximately 80%–90% confluence. Fibroblasts up to passage 3 identified by fibroblast specific protein 1 (FSP-1), vimentin, α-SMA, CD31 and Troponin T immunofluorescence staining (sup Fig. 1) were used in subsequent studies.

### MSCs isolation and culture

Wild type C57BL/6, leptin deficient ob/ob, and leptin receptor deficiet db/db (all with C57BL/6 background) used for MSC isolation were purchased from Model Animal Research Center of Nanjing University (Nanjing, China). Mouse MSCs were isolated from bone marrow of 4–5 week old wild type and ob/ob mice. Bone marrow extracted from the femur and tibia was flushed with Dulbecco's modified Eagle's medium: Nutrient Mixture F-12 (DMEM/F12, 100 U/mL penicillin G and 100 mg/mL streptomycin; Gibco, Carlsbad, CA, USA). After centrifugation, the cells were further cultured in DMEM containing 10% fetal bovine serum (FBS, Gibco) at 37°C and 5% CO2. After 24 hours, non-adherent cells were discarded, and adherent cells were washed with phosphate-buffered saline solution (PBS). Fresh complete medium was added and replaced every 3 days. Each primary culture was subcultured 1∶2 when MSCs grew to approximately 80%–90% confluence. After 3–5 passages, MSCs were characterized for their surface antigen profiling by Flow Cytometry as described previously.

### Hypoxia preconditioning protocol

Fresh complete medium was added to cell culture before hypoxia. Hypoxia treatment was achieved with a ProOx-C-chamber system (Biospherix, Redfield, NY) for 24 hours. The oxygen concentration in the chamber was maintained at 0.5%, with a residual gas mixture composed of 5% carbon dioxide and balanced nitrogen.

### Co-culture assay

Cardiac fibroblast activation was induced by culturing under hypoxia for 24 hrs. MSCs^WT^ and MSC^ob/ob^ plated in an insert was preconditioned by either hypoxia or normoxia for 24 hrs. Then CFs and MSCs were co-cultured in two chambers separated by a semipermeable membrane with 3 µm pore which will prevent cells contact but allow other materials exchange. MSCs were cultured in the upper inserts chamber, while CFs were planted in the lower chamber. After 24 hour co-culture, the inserts were removed, and CFs were collected for subsequent experiments.

### Real-time reverse-transcription polymerase chain reaction

Total cellular RNA from CFs after normoxia culture, hypoxia and TGF-beta treatment was extracted by Trizol Reagent (Invitrogen) according to the manufacturer's protocol. Total RNA (1 µg) was reverse transcribed with oligo (dT) 18 and M-MLV reverse transcriptase (TAKARA, Japan). The resulting cDNA mixture (1 µl) was employed for a PCR program of 40 cycles of melting (10 s at 95°C) and annealing (32 s at 60°C) with SYBR Premix Ex Taq (TAKARA) in Step One Plus Real-Time PCR System (Applied Biosystems, Foster City, CA, USA). Primers used were α-SMA Left (CTGACAGAGGCACCACTGAA), α-SMA Right (CATCTCCAGAGTCCAGCACA). Data were analyzed by the 2^−ΔΔCt^ using β-actin as a reference gene.

### Western blot analysis

Whole-cell protein from co-cultured CFs was extracted by 2× SDS sample buffer (80 µl per well of 6-well plate). The cells were immediately scraped off the plate and transferred to a microcentrifuge tube on ice, heated at 95°C for 20 min. 5 µl of the cell protein extracts were electrophoresed in 12% sodium dodecyl sulfate polyacrylamide gel electrophoresis (SDS-PAGE), and transferred onto a 0.45 µm Polyvinylidene fluoride Immobilon-P transfer membrane (Millipore, Billerica, MA, USA) using a transblot apparatus (Bio-Rad). Membranes were blocked with 5% Skim Milk PBS for one hour at room temperature followed by 4°C overnight incubation with primary antibodies (α-SMA, SM-22α, collagen I and α-Tublin: Abcam, Cambridge, MA, USA; phosphor-Smad2: Cell Signaling Technology, Danvers, MA, USA; TGF-β1 and β-actin: Santa Cruz Biotechnology, Santa Cruz, CA, USA). After washing three times with 0.1% Tween-20 PBS, these membranes were incubated with appropriate horseradish peroxide–conjugated secondary antibodies for 1 hour at room temperature, and detected with Immobilon Western Chemiluminescent HRP Substrate (Millipore). β-actin and α-Tublin was used as a reference, analyzed by means of Image-lab analysis software (NIH, Bethesda, MD, USA).

### Immunofluorescence staining of Cardiac fibroblast

Following treatment, cardiac fibroblasts were washed in PBS, fixed with 10% formaldehyde solution 10 min at room temperature, and permeabilized with 0.1% Triton X-100 PBS 10 min at room temperature. Then cells were blocked in 5% BSA solution at room temperature followed by 4°C overnight incubation with primary antibodies (Vimentin, a-SMA, Fibroblast specific protein 1, Troponin T, CD31 and MRTF-A: Abcam, Cambridge, MA, USA). After washing three times with 0.1% Tween-20 PBS, these cells were incubated with appropriate fluorescein–conjugated secondary antibodies (Santa Cruz Biotechnology) for 2 hours at room temperature, followed with nuclear staining by Hoechst 33258 pentahydrate 1 µg/ml (Invitrogen, Eugene, Oregon, USA). The fluorescence was examined and photographed using Leica fluorescence microscope.

### Picrosirius red staining

Following treatment, cardiac fibroblasts were fixed in methanol −20°C overnight, and incubated in 0.1% Picrosirius red staining solution (Sigma-Aldrich, France) as per manufacturer's instructions. Picrosirius red was solubilized in 0.1N sodium hydroxide and the optical density was read at 540 nm (IMARK, Bio-Rad).

### Myocardial infarction model and cell transplantation

Wild type (C57BL/6, 8–10-week old, 20–25 g weight) mice were anesthetized by intraperitoneal injection of 4% chloral hydrate (4 mg/kg) ventilated via tracheal intubations connected to a rodent ventilator, MI was induced by permanent ligation of the left anterior descending coronary artery with 8–0 silk. Before transplantation, MSCs were lentivirally transduced with CMV-green fluorescent protein (GFP). Cell suspensions in 20–25 µl PBS, normoxia or hypoxia preconditioned MSCs (2×10^5^ cells/mice) or PBS were intramyocardial injected into the MI border zone just after coronary artery ligation by 5 point. The hearts were harvested 7 days and 28 days after infarction and the infarcted left ventricles (LV) were used for subsequent experiment (n>5).

### Masson trichrome staining

At day 7 and 28 after cell injection, the infarcted size was measured by Masson trichrome staining. Frozen tissue sections of heart tissues were stained with Masson's trichrome kit (Maixin. bio, Fuzhou, Fujian, China). Infarct area and total LV area were measured using Image Pro software and expressed as percentage of infarct size.

### Immunofluorescence staining of heart tissue

Heart tissues obtained seven days post-MI were dehydrated in 30% sucrose PBS solution and embedded in Tissue-Tek OCT compound (Sakura Finetek USA, Inc., Torrance, CA, USA) and snap frozen in drikold. Frozen tissue sections (6.0 µm thick) were fixed in 4% paraformaldehyde, permeabilized in 0.2% Triton X-100, blocked with 5% goat serum, followed by 4°C overnight incubation with primary antibodies (Collagen I: ab 292 Abcam, Cambridge, MA, USA) followed by incubation with respective secondary antibodies. After three time washing with 0.1% Tween-20 PBS, frozen slide were incubated with appropriate fluorescein–conjugated secondary antibodies (Santa Cruz Biotechnology) for 2 hours at room temperature, followed with nuclear staining by Hoechst 33258 pentahydrate 1 µg/ml (Invitrogen, Eugene, Oregon, USA). The fluorescence was examined and photographed using Leica fluorescence microscope.

### Statistical analysis

All data are presented as mean ± SEM. Differences between 2 groups were analyzed with two-tailed t-test. Multiple comparisons were done by one-way ANOVA using SPSS 17.0 statistical software. Statistical significance was defined as P<0.05.

## Supporting Information

Figure S1 **Characterization of cardiac fibroblast.** Immunofluorescence staining of Vimentin, Fibroblast specific protein-1, α-SMA, CD31, Troponon T and DAPI has done in isolated cardiac fibroblasts. CFs expressed Vimentin and FSP-1, and did not expressα-SMA, CD31 and Troponon T.
(DOCX)

## References

[1] HuX, YuSP, FraserJL, LuZ, OgleME, et al (2008) Transplantation of hypoxia-preconditioned mesenchymal stem cells improves infarcted heart function via enhanced survival of implanted cells and angiogenesis. J Thorac Cardiovasc Surg 135: 799–808.1837475910.1016/j.jtcvs.2007.07.071

[2] ElnakishMT, KuppusamyP, KhanM (2013) Stem cell transplantation as a therapy for cardiac fibrosis. J Pathol 229: 347–354.2301189410.1002/path.4111

[3] HuXY, WangWX, YuMJ, LiuXB, WuRR, et al (2011) Tongxinluo promotes mesenchymal stem cell tube formation in vitro. J Zhejiang Univ Sci B 12: 644–651.2179680510.1631/jzus.B1101005PMC3150718

[4] SegersVF, LeeRT (2008) Stem-cell therapy for cardiac disease. Nature 451: 937–942.1828818310.1038/nature06800

[5] DaiW, HaleSL, MartinBJ, KuangJQ, DowJS, et al (2005) Allogeneic mesenchymal stem cell transplantation in postinfarcted rat myocardium: short- and long-term effects. Circulation 112: 214–223.1599867310.1161/CIRCULATIONAHA.104.527937

[6] OhnishiS, SumiyoshiH, KitamuraS, NagayaN (2007) Mesenchymal stem cells attenuate cardiac fibroblast proliferation and collagen synthesis through paracrine actions. FEBS Lett 581: 3961–3966.1766272010.1016/j.febslet.2007.07.028

[7] ZhangZ, WangJA, XuY, JiangZ, WuR, et al (2013) Menstrual blood derived mesenchymal cells ameliorate cardiac fibrosis via inhibition of endothelial to mesenchymal transition in myocardial infarction. Int J Cardiol 168: 1711–1714.2360840210.1016/j.ijcard.2013.03.126

[8] van den BorneSW, DiezJ, BlankesteijnWM, VerjansJ, HofstraL, et al (2010) Myocardial remodeling after infarction: the role of myofibroblasts. Nat Rev Cardiol 7: 30–37.1994942610.1038/nrcardio.2009.199

[9] BujakM, FrangogiannisNG (2007) The role of TGF-beta signaling in myocardial infarction and cardiac remodeling. Cardiovasc Res 74: 184–195.1710983710.1016/j.cardiores.2006.10.002PMC1924687

[10] LeaskA (2010) Potential Therapeutic Targets for Cardiac Fibrosis: TGF, Angiotensin, Endothelin, CCN2, and PDGF, Partners in Fibroblast Activation. Circ Res 106: 1675–1680.2053868910.1161/CIRCRESAHA.110.217737

[11] VelasquezLS, SutherlandLB, LiuZ, GrinnellF, KammKE, et al (2013) Activation of MRTF-A-dependent gene expression with a small molecule promotes myofibroblast differentiation and wound healing. Proc Natl Acad Sci U S A 110: 16850–16855.2408209510.1073/pnas.1316764110PMC3801009

[12] SmallEM (2012) The actin-MRTF-SRF gene regulatory axis and myofibroblast differentiation. J Cardiovasc Transl Res 5: 794–804.2289875110.1007/s12265-012-9397-0

[13] Martinez-MartinezE, Jurado-LopezR, Valero-MunozM, BartolomeMV, BallesterosS, et al (2014) Leptin induces cardiac fibrosis through galectin-3, mTOR and oxidative stress: potential role in obesity. J Hypertens 10.1097/HJH.000000000000014924695395

[14] LiP, WangD, LucasJ, OparilS, XingD, et al (2008) Atrial natriuretic peptide inhibits transforming growth factor beta-induced Smad signaling and myofibroblast transformation in mouse cardiac fibroblasts. Circ Res 102: 185–192.1799188410.1161/CIRCRESAHA.107.157677

[15] DavisJ, MolkentinJD (2013) Myofibroblasts: Trust your heart and let fate decide. J Mol Cell Cardiol 10.1016/j.yjmcc.2013.10.019PMC399585524189039

[16] StenmarkKR, GerasimovskayaE, NemenoffRA, DasM (2002) Hypoxic activation of adventitial fibroblasts: role in vascular remodeling. Chest 122: 326S–334S.1247581010.1378/chest.122.6_suppl.326s

[17] OberringerM, MeinsC, BubelM, PohlemannT (2008) In vitro wounding: effects of hypoxia and transforming growth factor beta1 on proliferation, migration and myofibroblastic differentiation in an endothelial cell-fibroblast co-culture model. J Mol Histol 39: 37–47.1778657310.1007/s10735-007-9124-3

[18] MoonYM, KangHJ, ChoJS, ParkIH, LeeHM (2012) Nox4 mediates hypoxia-stimulated myofibroblast differentiation in nasal polyp-derived fibroblasts. Int Arch Allergy Immunol 159: 399–409.2284674410.1159/000337658

[19] ShortM, NemenoffRA, ZawadaWM, StenmarkKR, DasM (2004) Hypoxia induces differentiation of pulmonary artery adventitial fibroblasts into myofibroblasts. Am J Physiol Cell Physiol 286: C416–425.1456158910.1152/ajpcell.00169.2003

[20] HuX, WuR, ShehadehLA, ZhouQ, JiangC, et al (2014) Severe Hypoxia Exerts Parallel and Cell-specific Regulation of Gene Expression and Alternative Splicing in Human Mesenchymal Stem CellsMesenchymal Stem Cells. BMC Genomics In press.10.1186/1471-2164-15-303PMC423450224758227

[21] ShindeAV, FrangogiannisNG (2013) Fibroblasts in myocardial infarction: A role in inflammation and repair. J Mol Cell Cardiol 10.1016/j.yjmcc.2013.11.015PMC399582024321195

[22] DobaczewskiM, Gonzalez-QuesadaC, FrangogiannisNG (2010) The extracellular matrix as a modulator of the inflammatory and reparative response following myocardial infarction. J Mol Cell Cardiol 48: 504–511.1963165310.1016/j.yjmcc.2009.07.015PMC2824059

[23] MyersMG, CowleyMA, MunzbergH (2008) Mechanisms of leptin action and leptin resistance. Annu Rev Physiol 70: 537–556.1793760110.1146/annurev.physiol.70.113006.100707

[24] Martinez-MartinezE, MianaM, Jurado-LopezR, BartolomeMV, NetoFV, et al (2014) The potential role of leptin in the vascular remodeling associated with obesity. Int J Obes (Lond) 10.1038/ijo.2014.3724583853

[25] YamaguchiY, MannDM, RuoslahtiE (1990) Negative regulation of transforming growth factor-beta by the proteoglycan decorin. Nature 346: 281–284.237459410.1038/346281a0

[26] LiL, OkadaH, TakemuraG, KosaiK, KanamoriH, et al (2009) Postinfarction gene therapy with adenoviral vector expressing decorin mitigates cardiac remodeling and dysfunction. Am J Physiol Heart Circ Physiol 297: H1504–1513.1968418910.1152/ajpheart.00194.2009

[27] WolpeSD, SherryB, JuersD, DavatelisG, YurtRW, et al (1989) Identification and characterization of macrophage inflammatory protein 2. Proc Natl Acad Sci U S A 86: 612–616.264311910.1073/pnas.86.2.612PMC286522

[28] HohBL, HosakaK, DownesDP, NowickiKW, FernandezCE, et al (2011) Monocyte chemotactic protein-1 promotes inflammatory vascular repair of murine carotid aneurysms via a macrophage inflammatory protein-1alpha and macrophage inflammatory protein-2-dependent pathway. Circulation 124: 2243–2252.2200707410.1161/CIRCULATIONAHA.111.036061PMC3217188

[29] LeaskA (2007) TGFbeta, cardiac fibroblasts, and the fibrotic response. Cardiovasc Res 74: 207–212.1691961310.1016/j.cardiores.2006.07.012

[30] CriderBJ, RisingerGMJr, HaaksmaCJ, HowardEW, TomasekJJ (2011) Myocardin-related transcription factors A and B are key regulators of TGF-beta1-induced fibroblast to myofibroblast differentiation. J Invest Dermatol 131: 2378–2385.2177601010.1038/jid.2011.219PMC3199034

[31] SmallEM, ThatcherJE, SutherlandLB, KinoshitaH, GerardRD, et al (2010) Myocardin-related transcription factor-a controls myofibroblast activation and fibrosis in response to myocardial infarction. Circ Res 107: 294–304.2055882010.1161/CIRCRESAHA.110.223172PMC2921870

